RETRACTED

# Evaluation of low-cost custom made VAC therapy compared with conventional wound dressings in the treatment of non-healing lower limb ulcers in lower socio-economic group patients of Kashmir valley

**DOI:** 10.1186/s13018-015-0314-5

**Published:** 2015-12-10

**Authors:** Zameer Ali, Afshan Anjum, Lubna Khurshid, Hamayun Ahad, Saheel Maajid, Shabir Ahmad Dhar

**Affiliations:** Department of Orthopaedics SKIMS Medical College, Bemina, Srinagar, 190018 Jammu and Kashmir India

**Keywords:** DFU, VAC, NPWT

## Abstract

**Background:**

Negative-pressure wound therapy is a technique to achieve wound healing in patients with non-healing wounds of the lower limb; vacuum-assisted closure (VAC) therapy is a technique to accelerate the healing of non-healing ulcers that fail to heal on their own (primary healing) (Plast Reconstr Surg 117:193–209S, 2006).

Delayed wound healing or non-healing of ulcers is a significant health problem, particularly in older adults.

The efficacy of VAC dressings has been demonstrated in several randomized controlled studies, which have shown significantly faster wound healing rates compared to conventional wound therapy (Lancet 366:1704–10, 2005; J Wound Care 17:426–32, 2008). However, commercially available VAC is costly.

The aim of using custom made VAC was decided by our team due to lower socio-economic status of patients taken for study who could not have afforded charges of commercially available VAC unit.

**Objective:**

Objective was to evaluate VAC therapy compared with conventional dressings in the treatment of non-healing lower limb ulcers in lower socio-economic patients.

**Methods:**

Sixty patients of lower socio-economic status aged between 40 and 70 were prospectively studied for non-healing ulcers Wagner grade 2 or 3 and randomized into 2 groups. VAC dressing was kept for over a period of 2–7 weeks. Ulcers were treated until the wound closed spontaneously, surgically or until completion of the 50-day period, whichever was earlier.

**Results:**

By seventh week, discharge disappeared in 96 % in VAC and only 54 % in conventional dressing group.

Granulation tissue appeared in 100 % of patients in VAC group and only 63 % in conventional dressing group. The patients treated with VAC dressing in our study showed comparable wound reduction capabilities with an average wound size reduction of 56 % in comparison to conventional dressing group which had average wound size reduction of 29 %.

Majority of wounds in VAC group got closed in 7 weeks. Patient satisfaction was excellent in the majority of patients in VAC group compared to those in conventional dressing group.

**Conclusion:**

The application of VAC™ had shown good results in our study.

RETRACTED

## Background

The purpose of this study is to share our experience with the vacuum-assisted closure (VAC) therapy compared with conventional wound dressings in the treatment of non-healing lower limb ulcers in lower socio-economic group patients. Negative-pressure wound therapy is a technique to achieve wound healing in patients with non-healing wounds of the lower limb; VAC therapy is a technique to accelerate the healing of non-healing ulcers that fail to heal on their own (primary healing) [1].

A mainstay of treatment of non-healing ulcers is meticulous debridement of all necrotic, devitalized and fibrous tissue, with a primary goal to obtain healing of ulcer and ultimately closure of wound. Management of non-healing ulcers differs in different institutions; hence, optimal treatment is ill-defined [2, 3, 4].

The vacuum-assisted closure (VAC®) device (KCI, San Antonio, TX) was pioneered by Dr. Louis Argenta and Dr Michael Morykwas in 1993 (Rosser et al. 2000). It is a development from the standard surgical procedure for treating non-healing ulcers, which uses controlled negative pressure using vacuum-assisted drainage to remove blood or serous fluid from wound site, to provide a drier surgical field and control blood flow (Thomas 2001) [5].

The US Food and Drug Administration (FDA) approved the use of VAC for the treatment of non-healing wounds in 1995. In January 2000, the approval was updated to include acute, sub-acute, chronic, and traumatic wounds (Mendez-Eastman 2001).

In VAC therapy, the application of topical negative pressure (vacuum) removes blood and serous fluid, reduces infection rates (closed/sealed system creates a hypoxic environment), further increasing localized blood flow, thereby supplying the wound with oxygen and nutrition to promote accelerated healing (vacuum therapy in wound management 2001, Genecov 1998).

Alternative names for VAC include topical negative pressure, sub-atmospheric pressure, sealed surface wound suction, vacuum sealing and foam suction dressing (vacuum therapy in wound management 2001).

Delayed wound healing or non-healing of ulcers is a significant health problem, particularly in older adults. Failure/prolongation of treatment of these ulcers is not only pain and suffering to patient but also to treating surgeon as well. Failure of the wound to heal also imposes social and financial burdens. Vacuum-assisted closure (VAC) therapy has been developed as an alternative to the standard forms of wound management, which incorporates the use of negative pressure to optimize conditions for wound healing [1–5].

A wound is considered to be chronic when it requires a prolonged time to heal, does not heal, or recurs after showing initial healing (Kranke et al. 2003). The prevalence of chronic wounds increases with age with a prevalence of 1.3 % in the Australian adult population, rising to 3.6 % for those aged 65 years and over (Rauchberger 2002). As age advances, there is a gradual decline in the function of sensory nerves that have an important role in tissue repair (Flicker 1996).

RETRACTED

Lower limb ulcers affect 10–25 % of diabetic patients. Management of a diabetic foot ulcer is often a challenging problem. Healing of these ulcers often takes a long time and may need one or more debridement. The treatment of such ulcers, therefore, needs time with a prolonged hospital stay, intensive wound management, and high hospitalization costs [1, 6].

The optimal topical therapy for non-healing lower limb ulcers remains poorly defined. Saline-moistened gauze has been the standard method; however, it has been difficult to continuously maintain a moist wound environment with these dressings. Subsequently, various dressing techniques like growth factors, hydrocolloid wound gels, enzymatic debridement compounds, hyperbaric oxygen therapy, cultured skin substitutes, and other wound therapies have been advocated. All of these therapies are expensive and time consuming also, there is little scientific evidence to support their efficacy [1, 7, 8].

Results of VAC indicate that VAC therapy is less costly and more effective than traditional dressings. Despite advances in management of ulcers, healing of difficult wound continues to be a challenge. NPWT is a technique that uses foam dressing that is put inside the wound cavity and applying negative pressure of 120–130 mmHg [2, 6].

Over the years, several advanced wound care products have been developed, all with the aim of achieving wound bed optimization for eventual wound closure. Negative pressure wound therapy (NPWT) using the vacuum-assisted closure (VAC) has shown good results in the management of non-healing ulcers. VAC therapy has gained increasing popularity for the treatment of chronic and complex wounds. The NPWT has been shown to accelerate wound healing by reducing local tissue edema, promoting granulation tissue formation, increasing local blood flow, and decreasing bacterial burden in both animal and clinical studies [2, 5]. The efficacy of VAC dressings has been demonstrated in several randomized controlled studies, which have shown significantly faster wound healing rates compared to conventional wound therapy [3, 9].

The studies conducted on the role of NPWT for the management of non-healing lower limb ulcers are limited.

Therefore, we conducted a prospective case-control study to evaluate the role of VAC in comparison to conventional dressings in the healing of non-healing ulcers in lower socio-economic group patients (Figs. 1, 2 and 3).

RETRACTED

**Fig. 1:** Instruments required for VAC. Dressing set, suction tube with side pores, Ioban and sterile foam

**Fig. 2:** VAC applied to patient with non-healing ulcer following fasciotomy. Look at the wrinkles on Ioban following active suctioning of VAC. A well-covered foam and mesentery around suctioning tube

**Fig. 3:** In-hospital suctioning unit for VAC. Pressure gauge for monitoring VAC pressure

The aim of using custom made VAC was decided by our team due to lower socio-economic status of patients taken for study who could not have afforded charges of commercially available VAC unit.

## Material and methods

This study was prospective case-control series which was conducted by Postgraduate Department of Orthopaedics SKIMS Medical College Hospital Srinagar which is a tertiary care hospital. Our study was conducted between February 2014 and March 2015, 60 patients were treated for non-healing lower limb ulcers Wagner [10] grade 2 or 3. Ulcers were graded by Wagner system of grading. It was a randomized case-control study. The study population was made up of 30 male subjects and 30 female subjects with a mean age of 60 years (range, 40–70 years) (Tables 1 and 2).

**Table 1:** Age distribution of patients

GROUP	Age group in years	Mean age
VAC group	45–70	56.4
Conventional dressing group	40–64	52.2

**Table 2:** Gender distribution of patients

Group	Total	Males	Females
VAC group	30	14	16
Conventional dressing group	30	18	12

The study population included patients with non-healing lower limb ulcers admitted in our hospital with age range between 40 and 70 years were randomized either to group A (patients treated with VAC) or group B (patients treated with conventional dressings), with an equal number of patients in each group (*n* = 30) (Figs. 4 and 5). VAC dressing was kept for over a period of 2–7 weeks. Ulcers were treated until the wound closed spontaneously, surgically or until completion of the 50 day period, whichever was earlier. After wound closure, patients were followed on a regular basis. Patients who were discharged from the hospital after wound closure were followed twice weekly, then weekly, followed by every 2 weeks, and then monthly. Follow-up was done for up to 6 months. Treatment success was defined as wound closure within a period of 7 weeks.

**Fig. 4:** Gender distribution of patients in VAC group

**Fig. 5:** Gender distribution in conventional dressing group

The VAC device consisted of open-pore foam (reticulated polyurethane or polyvinyl alcohol) dressings cut to the shape of the wound and a vacuum unit providing either continuous or intermittent negative pressure.

RETRACTED

A detailed history, clinical examination and relevant investigations were performed in all patients. A written informed consent was obtained from all the patients in the study. Institutional ethical committee of our hospital gave approval for the study.

All the patients with non-healing ulcers included in the study, irrespective of group assigned, underwent initial surgical debridement. Later, wounds were treated with multiple irrigations with saline and minor debridement to remove slough or necrotic tissue when needed.

Preparation of wound was done in all patients in study.

- Step 1: preparation of wound bed
  Old dressing from the wound was removed and discarded. If required, a culture swab for microbiology was taken before wound irrigation with normal saline.
  Surface slough or necrotic tissue was surgically removed (minor surgical debridement) and adequate haemostasis achieved. Skin around ulcer was cleaned with spirit (Fig. 6).

**Fig. 6:** Non-healing stump after injury due to RTA. Stump could not be closed by routine daily dressing. Patient was referred to our institute from a peripheral hospital
- Step 2: foam placement
  Sterile, foam dressing was gently placed into the wound cavity to provide an even distribution of negative pressure over the entire wound bed to aid in wound healing (vacuum therapy in wound management 2001). There are two different types of foam available, black (applied into the wound) or pink foam (applied over the wound) (vacuum therapy in wound management 2001). Pink foam, polyurethane ether (PU), was used in our study. It has larger pores, is lighter, easily collapsible and hydrophobic with a pore size of 400 to 600 mm. It is used when the stimulation of granulation tissue and wound contraction is required. Suction tube was embedded in the foam (Figs. 7 and 15), which was then connected to a controlled vacuum pump with a gauge meter for pressure control. The amount of pressure applied ranged from 120 to 130 mmHg.

**Fig. 7:** Same patient after application of first VAC
- Placement of adhesive dressing for wound sealing
  The site is then sealed with an adhesive drape. In our study, we used iodine-impregnated adhesive dressing (Ioban, 3M) which covered at least 5 to 7 cm of surrounding healthy skin to ensure effective seal. Separate drapes were used for suction tube and covered at least 7 to 10 cm of tubing forming a mesentery like covering (Fig. 2).
- The application of negative pressure
  Controlled pressure is uniformly applied to all tissues on the inner surface of the wound (McCallon 2000) [9]. The foam dressing should compress in response to the negative pressure. The ideal pressure setting is 125 mmHg, but painful chronic wounds such as chronic leg ulcers are usually managed with lower therapeutic pressures of 50 to 75 mmHg. Higher pressures of 150 mmHg plus are used for large cavity wounds such as acute traumatic wounds, as they produce copious amounts of exudate (Collier 2003).

RETRACTED

Dressing was changed every 48 to 72 h or sooner if the wound was infected. (ASERNIP-S accelerated review of vacuum-assisted wound closure—Nov 2003) Care was taken when removing the adhesive drape to avoid irritating the peri-wound skin.

VAC technique removes oedema and increases vascularity; further helping in granulation tissue formation finally helps in wound healing. VAC therapy is a very good technique of treating non-healing or difficult-to-heal ulcers [8]. It has since been proposed that the application of sub-atmospheric pressure produces mechanical deformation or stress within the tissue resulting in protein and matrix molecule synthesis and enhanced angiogenesis [11].

Statistical analysis in our study was done by a statistician. All the data were entered in SPSS 14 and analyzed. Variables were analyzed and correlations were made by using the mean, average, and Pearson’s chi-square/Fisher’s exact test. Two groups were compared using Student’s *t* test. Results were expressed as *n* (%). *p* values of <0.05 was considered to be statistically significant.

### Inclusion criteria

Wounds treated with VAC in our study included:

- Diabetic foot ulcers.
- Pressure sores.
- Traumatic ulcers.
- Fasciotomy wounds.

And wounds post-drainage for abscess with exposure of deep structures such as tendon and fascia.

### Exclusion criteria

Following patients were excluded from study

- Patients with previous VAC therapy and those on other forms of advanced wound therapy like hyperbaric oxygen therapy, normothermic wound therapy, or growth factor therapy within 30 days of the study, start date were excluded.
- Patients on corticosteroids, immunosuppressive agents, or chemotherapeutic agents and patients with poorly controlled medical problems were also excluded from the study.
- Patients with malignancy in the wound, untreated osteomyelitis.
- Wounds with exposed arteries or veins.
- Patients on anticoagulants or with actively bleeding wounds.

## Results

A total of 60 patients who met the inclusion criteria were enrolled in the study. Patients were randomly assigned to either VAC group or conventional dressing group. Patients, either in VAC or conventional group, were matched for age, gender and grade of ulcer. After admission, patients were closely followed for signs of healing in both groups.

RETRACTED

All patients with diabetes were closely monitored for glycaemic control and routine endocrine consultations were sought in all the patients on daily basis. All patients were put on insulin for control of their blood sugars. Overall, lower doses of insulin were required to control hyperglycemia in VAC group as compared to conventional dressing group. Blood sugars were controlled within 1 week in VAC group as compared to 2–3 weeks in conventional dressing group.

In our study, the final point was taken as completely granulated wound, free of discharge or a wound ready for skin grafting or spontaneous healing by secondary intention.

Good protein diet was given to both groups as per hospital policy.

Age distribution of patients in VAC group was between 45 and 70 years with mean age of 56. While in conventional dressing group age, range was between 40 and 64 years with average of 52 years. Mean age of patients was slightly more in VAC group as compared to conventional dressing group.

Out of total, 60 patients studied each group received equal number of patients.

Majority of patients in VAC group were females as depicted in Fig. 4.

Majority of patients in conventional dressing group were males.

The average haemoglobin of all patients in VAC group was 10.4 g/dl. Minimum and maximum values were 8 and 13 g/dl. Two patients had haemoglobin of 8 g/dl and were transfused with packed cells.

Average haemoglobin of all patients in conventional dressing group was 11.2 g/dl. Minimum and maximum values were 9 and 14 g/dl.

Patients with anaemia were evaluated by general physician, and anaemic patients were started with iron supplementation, irrespective of group assigned.

Granulation tissue appeared in 73 % of patients in VAC group by the end of week 2 which further reached to 100 % by the end of week7 (Figs. 3 and 6). While in conventional dressing group, only 46 % of patients showed granulation tissue by the end of week 2 which further reached to 63 % by the end of week 7 (Figs. 8 and 9).

**Fig. 8:** After 4 weeks of VAC application: wound showed a significant improvement during the course of VAC treatment. The wound was dry with good granulation tissue and significant decrease in size in comparison to initial size of wound before application of VAC

**Fig. 9:** After 6 weeks of VAC application: further decrease in size of wound. Wound was dry with no signs of infection. During course of VAC application, gentle ROM for knee was advised to the patient

Granulation tissue was interpreted by the single observer in terms of gross appearance of ulcer.

Cultures were taken from the wound at the time of start of treatment, irrespective of group assigned.

RETRACTED

The microorganisms cultured from the ulcers in VAC group in decreasing order were *Pseudomonas aeruginosa* in 13 (43.3 %), staphylococcus aureus 10 (33 %), *Escherichia coli* 4 (13) *Acinetobacter baumannii* 3 (10 %) while that from the wounds in conventional dressing group were staphylococcus aureus 14 (46 %) *P. aeruginosa* in 12 (40 %) and *mixed flora* 4 (13.3 %). Antibiotics were given in terms of culture sensitivity reports.

Tables 3 and 4 shows Wound size decreased in 27 (90 %) patients in VAC group as compared to 19 (63 %) patients in conventional dressing group (Figs. 10 and 11).

**Table 3:** Frequency distribution of decrease in wound discharge in different groups

Group	Week 2 (%)	Week 7 (%)
VAC	18 (60 %)	29 (96 %)
Conventional dressing group	9 (30%)	16 (54%)

*p*value 0.04

Wounds were closely monitored for decrease in discharge with respect to time taken.

By week 2, wound discharge disappeared in 60 % of wounds in VAC group which further reached to 96 % in week 7 upon continuation of VAC.

By week 2 in conventional dressing group, wound discharge disappeared in 30 % which reached to 54 % in week 7 on continuation of dressings.

Above was statistically significant correlation with *p* value of less than 0.05.

The range of wound size in our study was from 11 to 21.6 cm^2^.

Average wound size in VAC group was 16 cm^2^ and average wound size in conventional dressing group was 13.6 cm^2^.

**Table 4:** Frequency distribution of appearance of granulation tissue in different groups

Group	Week 2 (%)	Week 7 (%)
VAC	22 (73)	30 (100)
Conventional dressing group	14 (46)	19 (63)

*p* value 0.01

**Fig. 10:** Follow-up of patient in OPD 1 month after discharge. Look at small callosity over the stump due to use of prosthesis

**Fig. 11:** Follow-up of patient in OPD 1 month after discharge. complete healing of ulcer is noted.

The patients treated with VAC dressing in our study showed comparable wound reduction capabilities with an average wound size reduction of 56 % in comparison to conventional dressing group which had average wound size reduction of 29 %.

One patient underwent ray amputation in VAC group as compared to three patients in conventional dressing group.

Eighteen patients in total were closed by split-thickness skin graft (STSG). Seven patients got closed spontaneously during the course of VAC treatment. Majority of the patients in VAC group were finally closed by split tissue skin grafting. STSG was done in routine theatre after ulcer was covered by granulation tissue and was devoid of discharge (Fig. 12).

**Fig. 12:** Descriptive statistics of final closure in VAC group

The majority of wounds were closed by a split-thickness skin graft in both groups (Tables 5 and 6).

RETRACTED

**Table 5:** Descriptive statistics of final closure in VAC group

VAC group	No. of patients	Final closure
Diabetic foot ulcers (DFU)	17	STSG (11), SC (4)
Pressure ulcers (PU)	4	STSG (1), SC (3)
Traumatic ulcers (TU)	6	STSG (4)
Post-fasciotomy wounds (PFW)	3	STSG (2)

**Table 6:** Descriptive statistics of final closure in conventional dressing group

Conventional dressing group	No. of patients	Final closure
Diabetic foot ulcers (DFU)	20	STSG (11), SC (2)
Pressure ulcers (PU)	3	STSG (2)
Traumatic ulcers (TU)	5	STSG (3)
Post-fasciotomy wound (PFW)	2	STSG (2)

Eighteen patients in total were closed by STSG. Two diabetic foot ulcers got closed spontaneously during the course of conventional saline moistened dressings (Fig. 13).

**Fig. 13:** Descriptive statistics of final closure in VAC group

The majority of wounds in VAC group 25 (83.3 %) were closed in 7 weeks as compared to only 20 (66 %) in conventional dressing group in 7 weeks (Fig. 14).

**Fig. 14:** Non-healing ulcer after Achilles tendon repair. Patient came to us with active discharge, with uncontrolled blood sugar. Wound culture was positive for pseudomonas. Initial minor debridement followed by copious lavage with saline was done in emergency OT. VAC was applied on first post-operative day

Patient satisfaction was excellent in the majority of patients in VAC group compared to those in conventional dressing group (Figs. 15 and 16)

**Fig. 15:** VAC in progress for the same patient. Wrinkles over Ioban are visible after application of negative pressure. Sugar got controlled after 5 days of application of VAC

**Fig. 16:** Healed ulcer after 4 weeks

.

No patient in our study reported discomfort with the application of pressures greater than 100 mmHg.

### Discussion

Our study was prospective case-control series which was conducted by Postgraduate Department of Orthopaedics SKIMS Medical College Hospital which is a tertiary care hospital situated in mountainous valley of Kashmir.

The ability of regular VAC dressings in promoting wound bed granulation and healing has been demonstrated in several studies. Application of VAC over the ulcer allows the arterioles to dilate, increasing local circulation, promoting angiogenesis, reduces bacterial burden and chronic interstitial wound fluid which finally leads to increased granulation tissue over the wound. Wound bed optimization is crucial in preventing ulcer complications and favours eventual wound closure either by split-tissue skin grafting or by secondary intention [3, 12].

In our study, we observed that the patients on VAC therapy had the early appearance of granulation tissue as compared to the patients treated by moist saline gauze dressings. Complete (100 %) granulation was achieved earlier and in a higher proportion of patients in VAC group as compared to conventional dressing group. Which is comparable to two large multicentric, randomized controlled trials conducted by Armstrong et al. [3] and Blume et al. [13]. They reported a median time of 42 and 56 days, respectively, for 76–100 % wound bed granulation using VAC dressings for average wound sizes of 22.3 and 13.5 cm^2^, respectively.

RETRACTED

In our study by week 2, wound discharge disappeared in 60 % of wounds in VAC group which further reached to 96 % in week 7 upon continuation of VAC in comparison to conventional dressing group; wound discharge disappeared in 30 % at 2 weeks which reached to 54 % in week 7 on continuation of dressings (this was statistically significant correlation with *p* value of 0.04).

Thus, rate of disappearance of wound discharge was faster in VAC group as compared to conventional dressing group, which was statistically significant (*p* < 0.04), similar to observations made by Prabhdeep SN, et al. [14, 15].

The range of wound size in our study was from 11 to 21.6 cm^2^ with average wound size in VAC group was 16 cm^2^ and average wound size in conventional dressing group was 13.6 cm^2^ which was comparable to study by McCallon [13, 9, 11].

In our study, wound size decreased in 27 (90 %) patients in VAC group as compared to 19 (63 %) patients in conventional dressing group. The results are comparable to the study conducted by Mullner et al.—a prospective trial involving 45 patients with soft tissue injuries including sacral pressure ulcers, acute traumatic soft tissue defects and infected soft tissue defects following rigid stabilisation of lower extremity fractures. They reported that in 38/45 patients (84 %), the use of the vacuum sealing technique following irrigation and debridement decreased the dimensions of the initial wound, thus facilitating healing time and the eradication of any pre-existing infection.

The patients treated with VAC dressing in our study showed comparable wound reduction capabilities with an average wound size reduction of 56 % in comparison to conventional dressing group which had wound size reduction of 29 %. These results are comparable to randomized controlled crossover trial by Eginton et al. [12] who achieved an average 59 % wound volume reduction in patients on VAC.

Another study conducted by McCallon et al. observed an average decrease of 28.4 % (±24.3) in wound size in the VAC group as compared to 9.5 % (±16.9) average decrease in wound size in the control group (treated by saline-moistened gauze dressings). Mark et al. had also observed that the wound volume and depth decreased significantly in VAC dressings as compared to moist gauze dressings [9, 16].

RETRACTED

Study conducted by M. Singh et al. reported gratifying results with manually operated vacuum devices. Singh et al. performed NPWT using Romovac or similar 18 Fr. drain. They described it to be a simple and effective method of NPWT which should benefit the larger population where the standard equipment is not available [10].

One patient underwent ray amputation in VAC group as compared to three patients in conventional dressing group. Numbers of amputations were lesser in VAC group. Our study was comparable to study conducted by Blume et al. While assessing the safety of VAC, he reported fewer numbers of secondary amputations in VAC-treated patients as compared to those treated by saline gauze dressings [13].

The majority of wounds in our patients were closed by a split-thickness skin graft in both groups.

Eighteen patients in total were closed by STSG. The majority of wounds in VAC group 25 (83.3 %) were closed in 7 weeks as compared to only 20 (66 %) in conventional dressing group in 7 weeks.

Our study is comparable to study conducted by Argenta LC et al. in their study of 296 wounds majority responded favorably to VAC treatment. Majority of patients needed STSG for coverage after wound was free from discharge and had good granulation tissue coverage they authors concluded that VAC is an extremely efficacious modality for treating chronic and difficult to heal wounds.

## Conclusion

The application of VAC™ as modality of treatment for non-healing ulcers supports wound conditioning and facilitates the definitive wound care.

The VAC dressing was found to be effective in the treatment of non-healing lower limb ulcers. It promotes wound area reduction, wound bed granulation, and achieves microbial clearance.

Although, most studies on VAC therapy reveal good results and better healing of ulcers than standard methods. More rigorous studies with larger sample sizes assessing the use of VAC therapy on different types of wounds are required.

With proper training to ensure appropriate and competent use, VAC is simple to use and appears to be a promising alternative for the management of various wound types.

## References

[1] Brem H, Sheehan P, Rosenberg HJ, Schneider JS, Boulton AJ (2006). Evidence-based protocol for diabetic foot ulcers. Plast Reconstr Surg.

[2] Argenta LC, Morykwas MJ (1997). V.A.C.uum-assisted closure: a new method for wound control and treatment: clinical experience. Ann Plast Surg.

[3] Armstrong DG, Lavery LA (2005). Diabetic Foot Study Consortium. Negative pressure wound therapy after partial diabetic foot amputation: a multicentre, randomised controlled trial. Lancet.

RETRACTED

[4] Eginton MT, Brown KR, Seabrook GR, Towne JB, Cambria RA (2003). A prospective randomized evaluation of negative-pressure wound dressings for diabetic foot wounds. Ann Vasc Surg.

[5] Morykwas MJ, Argenta LC, Shelton-Brown EI, McGuirt W (1997). V.A.C.uum-assisted closure: a new method for wound control and treatment: animal studies and basic foundation. Ann Plast Surg.

[6] American Diabetes Association (1999). Consensus development conference on diabetic foot wound care. Diabetes Care.

[7] Ramanujam CL, Stapleton JJ, Zgonis T (2013). Negative-pressure wound therapy in the management of diabetic Charcot foot and ankle wounds. Diabet Foot Ankle.

[8] Fabian TS, Kaufman HJ, Lett ED, Thomas JB, Rawl DK, Lewis PL (2000). The evaluation of subatmospheric pressure and hyperbaric oxygen in ischemic full-thickness wound healing. Am Surg.

[9] White R, McIntosh C (2008). Topical therapies for diabetic foot ulcers: standard treatments. J Wound Care.

[10] Mullner T, Mrkonjic L, Kwasny O, Vecsei V (1997). The use of negative pressure to promote the healing of tissue defects: a clinical trial using the vacuum sealing technique. Br J Plast Surg.

[11] Singh M, Singh R, Singh S, Pandey V, Singh D (2009). Vacuum assisted closure in wound management-Poor man's VAC©. Internet J Plast Surg.

[12] Mark TE, Kellie RB, Gary RS, Jonathan BT, Robert AC (2003). Prospective randomized evaluation of negative–pressure wound dressing for diabetic foot wounds. Ann Vasc Surg.

[13] Blume PA, Walters J, Payne W, Ayala J, Lantis J (2008). Comparison of negative pressure wound therapy using V.A.C.uum-assisted closure with advanced moist wound therapy in the treatment of diabetic foot ulcers: a multicenter randomized controlled trial. Diabetes Care.

[14] Wagner FW (1981). The dysvascular foot: a system for diagnosis and treatment. Foot Ankle.

[15] Peycru T, Tardat E, Lepront D, Schwartz A, Jarry J, Durand-Dastes F (2008). Vacuum-assisted abdominal closure in the critically ill patient. The poor man’s VAC]. [Article in French] (Paris). J Chir.

[16] Prabhdeep SN, Sanjeev KU, Ramneesh G, Kuljyot B, Shirin G (2011). Role of negative pressure wound therapy in healing of diabetic foot ulcers. J Surg Tech Case Rep.

